The article "Xianglian Pill Suppresses Inflammation and Protects Intestinal Epithelial Barrier by Promoting Autophagy in DSS Induced Ulcerative Colitis Mice" was retracted in 2023. Reasons: original data or images not available; unreliable results or conclusions; concerns about the data.

# Xianglian Pill Suppresses Inflammation and Protects Intestinal Epithelial Barrier by Promoting Autophagy in DSS Induced Ulcerative Colitis Mice

**DOI:** 10.3389/fphar.2020.594847

**Published:** 2021-01-27

**Authors:** Bingyu Wang, Zhiqiang Gong, Jingyu Zhan, Lei Yang, Quanyu Zhou, Xingxing Yuan

**Affiliations:** ^1^ Department of Gastroenterology, Heilongjiang Academy of Traditional Chinese Medicine, Harbin, China; ^2^ College of Chemistry and Chemical Engineering, Guangxi University for Nationalities, Nanning, China; ^3^ Department of Emergency, Heilongjiang Academy of Traditional Chinese Medicine, Harbin, China

**Keywords:** Xianglian pill, ulcerative colitis, inflammation, intestinal epithelial barrier, autophagy

## Abstract

Xianglian pill (XLP) is a typical traditional Chinese herbal medicine prescription composed of Coptidis Rhizoma and Aucklandiae Radix. It has been used to treat gastrointestinal disease for centuries. In the present study, the potential mechanisms of XLP in the treatment of ulcerative colitis (UC) were predicted by integrative pharmacology-based approach. Then, the main compounds of XLP were detected by liquid chromatography-mass spectrometry (LC-MS/MS). Finally, we verified the mechanism of XLP in the treatment of UC in a dextran sulfate sodium (DSS) model. C57BL/6 mice were randomly divided into the control group, DSS group, 5-aminosalicylic acid (5-ASA) group which was used as the positive drug control, XLP low, medium, and high dose group, with 10 mice per group. Except for the control group, acute colitis model was induced in the other mice by administering 3% DSS for consecutive 7 days. Mice in 5-ASA and XLP groups were administered with 5-ASA (50 mg/kg) or XLP (0.8, 1.6, 3.2 g/kg) via oral gavage once per day respectively. Body wight and disease activity index were assay during drug intervention. On day 8, all animals in this experiment were sacrificed and colon tissues were collected for analysis after measurement of the length. The results showed that XLP alleviate DSS -induced acute colitis in mice, including inhibition the secretion of pro-inflammatory cytokines, repairing the dysfunction of intestinal epithelial barrier, enhanced autophagy, and blocked the activation of PI3K/Akt/mTOR pathway. Furthermore, inhibiting autophagy by 3-methyladenine attenuated the protective effects of XLP on colitis. The underlying mechanism may be that Xianglian pill promote autophagy by blocking the activation of PI3K/Akt/mTOR signaling pathway.

## Introduction

Ulcerative colitis (UC) is an idiopathic inflammatory disorder of the large intestine that starting with mucosal inflammation in the rectum and often extending proximally to involve additional areas of the colon (Rubin et al., 2019). It is one of the two major manifestations of inflammatory bowel disease (IBD), and characterized by imbalanced of cytokines and immune dysfunction and unresolved inflammation associated with intestinal mucosa (Sairenji et al., 2017). Usually, patients with UC present with bloody diarrhea, abdominal pain, fecal urgency, and tenesmus, with an increasing incidence worldwide (Molodecky et al., 2012). Nearly 286 cases per 100,000 population in the United States and 505 of 100,000 in Europe are affected by this condition and many more globally (Ungaro et al., 2017). Less data is available from developing countries; however, recognition of ulcerative colitis is increasing in Asia, the Middle East, and South America (Sood et al., 2003; Tozun et al., 2009; Victoria et al., 2009).

Despite huge progress have been made in understanding its mechanism in recent years, its exact pathogenesis is still unclear. The pathogenesis of UC is multifactorial, involving epithelial barrier defect, excessive inflammatory response, immune response disorder, genetic predisposition, and environmental factors. Among these, intestinal epithelial barrier function plays a pivotal role in the occurrence and development of UC (Parikh et al., 2019). The epithelial barrier comprises specialized cells with diverse functions that emerge from stem cells at the crypt base, which form the first barrier to resist the harsh environment. Tight junctions of epithelial cells are composed of transmembrane proteins (such as claudins and occludins) and auxiliary proteins (zonula occludens, ZOs), which are used to prevent the spread of pathogens and harmful antigens on the epithelium (Fasano, 2011). Recent studies have shown that UC submucosal inflammation affects the integrity of epithelial barrier structure, which leads to the change of intestinal permeability, thus promoting the abnormal immune response (Chang et al., 2017). Therefore, to enhance the function of intestinal mucosal barrier may be a treatment for UC.

The effectiveness, safety and quality of traditional Chinese medicine (TCM) related products have attracted worldwide attention. Xianglian pill (XLP), a typical TCM prescription composed of Huanglian (Coptidis Rhizoma) and Muxiang (Aucklandiae Radix), have been used to treat gastrointestinal disease for centuries in TCM. Coptidis Rhizoma is derived from the dried roots of Coptis chinensis Franch. Previous studies have demonstrated that it has wide pharmacological activities, including anti-inflammatory, antidiarrheal, anti-cancer activities, and therapeutic potential on hypertension and diabetes (Sun et al., 2009; Chen et al., 2014; Lan et al., 2015; Li et al., 2019). Aucklandiae Radix is the dried root of Aucklandia costus Falc., which has been used as a medicinal material for digestive system disorders in TCM for centuries. It has been reported that the main active components of Aucklandiae Radix possessed anti-inflammatory, anti-bacterial, and anti-tumor activities. Previously, the therapeutic effects of Aucklandiae Radix on gastrointestinal function and smooth muscle spasm and on UC induced by DSS have been confirmed (Guo et al., 2014). To provide more evidence for the potential application of TCM prescription in UC therapy, an integrative pharmacology-based approach was employed to understand the effect of XLP on UC in the present study. This study is divided into three parts: 1) Predicting the target of XLP in the treatment of UC by bioinformatics, the bioinformatics workflow is shown in Figure 1A; 2) Analyzing the main components of XLP by liquid chromatography-mass spectrometry (LC-MS/MS); 3) Verifying the candidate target pathway of XLP in DSS induced UC mice model.

**FIGURE 1:** Study of Xianglian pill in the treatment of ulcerative colitis using integrative pharmacology-based approach. **(A)** The work flow of the study using an integrative pharmacology-based approach. **(B)** Disease gene-drug target network was constructed by Cytoscape software. **(C)** Results of the analysis of enriched GO biological processes. **(D)** Results of the analysis of enriched KEGG pathways.

## Materials and Methods

### Target Prediction and Network Analysis

The active components and targets of Coptidis Rhizoma and Aucklandiae Radix were obtained by searching the Encyclopedia of Traditional Chinese Medicine (ETCM, http://www.nrc.ac.cn:9090/ETCM/) (Xu et al., 2019), this platform combines a variety of authoritative algorithms, including physical and chemical properties, drug-forming evaluations, absorption and distribution of metabolic excretion index scores, target prediction, etc. Drug target (Drugbank, http://www.drugbank.ca, version: 5.1.7) and GeneCards (https://www.genecards.org/) databases were used to search and screen the target genes of UC, and the target genes were combined to eliminate the repeated disease targets. Finally, the disease gene-drug target network was constructed by extracting the intersecting target genes.

### GO and Pathway Enrichment

By using the online Database for Annotation, Visualization and Integrated Discovery (DAVID, https://david.ncifcrf.gov/, version 6.8), the XLP candidate targets against UC were analyzed by determining the related GO biological processes and signaling pathways that were enriched in the KEGG (http://www.genome.jp/kegg/, last updated on October 16, 2012).

### Materials

XLP was purchased from the Hubei Xianglian Pharmaceutical Co., Ltd. (Z42020398, Hubei, China, the compositions were shown in Table 1). Standard solutions of berberine, jatrorrhizine, costunolide, coptisine, and palmatine were purchased from Yuanye Bio-Technology Co., Ltd (Shanghai, China, cat# B21449, B21451, B20891, B21438, B21433). DSS (36,000–50,000 MW) was purchased from MP Biomedicals (Santa Ana, CA, United States, cat# 160110). 5-aminosalicylic acid (5-ASA) was purchased from Sigma-Aldrich (St. Louis, MO, United States, cat#A79809). 3-methyladenine (3-MA) was purchased from Selleck (Huston, TX, United States, cat#S2767).

**TABLE 1:** Composition of Xianglian pill.

Chinese name	Latin name	English name	Quantity (ratio in dry weight)
Huanglian	Coptis chinensis Franch	Coptidis Rhizoma	4
Muxiang	Aucklandia costus Falc	Aucklandiae Radix	1

### Analysis of Xianglian Pills by Liquid Chromatography-Mass Spectrometry

The dried sample of XLP powder were ground to pass through a 60-mesh sieve. The sample (0.1 g) was suspended in methanol (50 ml), and ultrasonic treatment for 30 min. The supernatant was diluted 160 times with methanol and centrifuged at 14,000 r/min for 10 min. The supernatant was then filtered through a 0.22 μm microporous membrane. Five standard stock solutions including berberine (0.26 mg/ml), jatrorrhizine (0.44 mg/ml), costunolide (0.22 mg/ml), coptisine (0.38 mg/ml), and palmatine (0.38 mg/ml) were individually prepared in methanol. The solution was then filtered through a 0.22 μm micropore membrane. Liquid Chromatography: Agilent Technologies 1260 series high pressure mixing pump (Boston, MA, United States) was used for liquid chromatography separation. Agilent EclipsePlus-C18 (2.1 mm inner diameter × 50 mm) 1.8 μm particle size column (Boston, MA, United States) was used with a mobile phase gradient of solvent A (water containing 0.1% formic acid): solvent B (acetonitrile) as 10:90. The elution time was 12 min. Mass Spectrometry: An AB Sciex QTRAP 4500 tandem mass spectrometer (Foster, CA, United States), operated with a Turbo-V Ion Spray source was used to obtain the Scheduled MRM determination (MRM-IDA-EPI). The optimized conditions were as follows: ion spray voltage, 5.5 kV; Ion Source gas 1, 55; Ion Source gas 2, 55; turbo temperature, 500°C; entrance potential, 10 V; and declustering potential (DP), 60 V. The collision gas pressure was set at 8.0 Arb and the curtain gas pressure at 30.0 Arb. The MRM transitions and the related optimized DP.

### The Establishment of Ulcerative Colitis Mice Model

C57BL/6 mice (male, 7–8 weeks old) were purchased from Beijing Vital River Laboratory Animal Technology Co., Ltd. (Beijing, China) (Production license number was SCXK Beijing, 2012–0001 and the Certificate No.11400700008581). After acclimatization for at least one week, sixty mice (weigh, 20–22 g) were randomly divided into six group: control group, DSS group, 5-ASA group, XLP low dose group, XLP medium dose group, and XLP high dose group, with 10 mice per group. Except for the control group, acute colitis model was induced in mice by administering 3% DSS dissolved in drinking water for consecutive 7 days as previously described (Qu et al., 2017). According to the conversion rate of clinical administration dose and experimental animals, the mice in 5-ASA group and XLP groups were administered with 5-ASA (50 mg/kg) or XLP (0.8, 1.6, 3.2 g/kg) via oral gavage once per day respectively. Mice in the control group and DSS group were given the same volume of saline. On day 8, all animals in this experiment were sacrificed and colon tissues were collected for analysis after measurement of the length. Experimental design and grouping were shown in Figure 2A.

**FIGURE 2:** Schematic diagram and analysis of main compounds of Xianglian pill. **(A)** Experimental design and grouping of the study. **(B)** Extracted Ion Chromatogram of five main chemical components in mixed standard stock solution. **(C)** Extracted lon chromatogram of five main chemical components in XLP solution. **(D)** Total lon chromatograms of five main chemical components in mixed standard stock solution. **(E)** Total lon chromatograms of five main chemical components in XLP solution.

### Disease Activity Index Assessment

Mice were monitored daily for body weight and stool consistency as well as the presence of gross blood in the feces from day 1 to day 7. The disease activity index (DAI) was calculated according to the well-established methods (Bang and Lichtenberger, 2016): 1) loss of body weight loss: 0 = none; 1 = 1–5%; 2 = 5–10%; 3 = 10–15%; 4 = over 15%; 2) stool consistency: 0 = normal; 2 = loose stools; 4 = diarrhea; 3) presence of gross bleeding or bloodstain: 0 = negative; 2 = positive; 4 = gross rectal bleeding.

### Histologic Analysis

The distal colonic tissues of mice were fixed in 4% paraformaldehyde and stained with hematoxylin and eosin (H&E, Jiancheng, Nanjing, China, cat#D006-1). Colonic histological tissues were observed under a light microscope (Olympus, Tokyo, Japan). Histological damage to the colon were calculated as previously described (Qu et al., 2017).

### Enzyme-Linked Immunosorbent Assay

Colons were weighed and homogenized, the lysate was centrifuged at 4°C for 15 min (12,000 g), and the supernatant was used for analyses. The levels of tumor necrosis factor (TNF)-α, interleukin (IL)-1β, IL-6, IL-8, IL-17, IFN (Interferon)-γ, myeloperoxidase (MPO), inducible nitric oxide synthetase (iNOS), and nitric oxide (NO) in colons were measured by corresponding ELISA kits (Meimian, Jiangsu, China, cat#MM-0132M2, MM-0040M2, MM-0163M2, MM-0123M2, MM-0170M2, MM-0182M2) and MPO, iNOS, NO assay kits (Jiancheng, Nanjing, China, cat#A044-1-1, A014-1-2, A013-2-1) following the manufacturer’s instructions.

### Western Blotting Analysis

Colon tissues were weighed and homogenized with cold RIPA lysis buffer (Beyotime, Jiangsu, China, cat#P0013B) supplemented with protease and phosphatase inhibitors on the ice. Subsequently, the homogenates were centrifugated at 4°C for 5 min (12,000 g), the supernatants were then collected and protein concentration was determined by using BCA protein assay kit (Beyotime, Jiangsu, China, cat#P0010S). 50 µg total protein from colon tissue in the lysate were then separated via SDS-PAGE and transferred onto a polyvinylidene fluoride (PVDF) membrane (Millipore, MA, United States) for 2 h by a wet transfer method. Thereafter, the membrane was blocked with 5% non-fat milk in TBST buffer for 2 h at room temperature, and incubated with primary antibodies at 4°C overnight. The primary antibodies from Cell Signaling Technology (Danvers, MA, United States, cat#13255, 13,663, 3495, 4257, 4060, 4691, 5536, 2983, 4970) or Abcam Technology Inc (Cambridge, MA, United States, cat#ab192890) including Claudin-1, ZO-1, Beclin-1, LC3B, PI3K, p-Akt, Akt, p-mTOR, mTOR, and β-actin antibodies (1:1000 dilution). After three times washed with TBST, the membrane was incubated with HRP-conjugated secondary antibody (1:1000 dilution, Beyotime, Jiangsu, China, cat#A0208) for 1 h at room temperature. After then, the labeled band were detected using an ECL kit (Beyotime, Shanghai, China, cat#P0018M). The signal intensity was detected by ImageJ software.

### Immunofluorescence Staining

Immunofluorescence staining were performed on paraffin sections of colon tissue. After dewaxing and rehydration, antigen retrieval was performed in sodium citrate buffer (pH 6.0) for 3 min by microwaving the sections. Sections were then blocked using 1% sheep serum in PBS for 1 h at room temperature and immunostained with primary antibodies overnight at 4°C. The primary antibodies from Cell Signaling Technology including Claudin-1 and ZO-1. Afterward, sections were washed by PBST and incubated with Alexa Fluor 594-conjugated IgG secondary antibody (1:1000 dilution, Abcam, MA, United States, cat#ab150116) for 2 h at room temperature, followed by counterstaining with DAPI (10 μg/ml) for 5 min, and mounted using antifade solution. Finally, sections were photographed under a fluorescence microscope (Olympus, Tokyo, Japan).

### Quantitative Real-Time PCR Analysis

Total RNA from colon tissues was extracted with Trizol reagent (Solarbio, Beijing, China, cat#R1100) according to the manufactures’ instructions. Then, the cDNA was obtained using reverse transcribe PrimeScript 1st Strand cDNA synthesis kit (TAKARA, Kyoto, Japan, cat#6210A). Real-time reverse-transcription polymerase chain reaction was carried out using SYBR Green qPCR Mix (Applied Biosystems, CA, United States cat#A25741) on a Roche LightCycler 480 (Roche, Switzerland). Forward and reverse primers of related genes were as shown in Table 2. The relative expression of the target genes was calculated by the 2^−ΔΔCT^ method with normalization to GAPDH mRNA.

**TABLE 2:** Primers used in quantitative real-time PCR reactions.

Gene	Forward primer (5′ to 3′)	Reverse primer (5′ to 3′)	Product length (bp)
Claudin-1	CGA​GCC​CTA​ATG​GTG​GTC​TC	GCA​AGA​CCT​GCC​ACG​ATG​AA	155
ZO-1	CGC​CTC​TGT​CCA​ACT​CTT​CTC​T	GGT​GTG​AAT​CGG​TTG​TAT​GCT​G	265
GAPDH	ATG​CAA​CGG​ATT​TGG​TCG​TAT	TCT​CCT​CCT​GGA​AGA​TGG​TG	211

### Transmission Electron Microscopy Analysis

A total of 1 cm^2^ sections of distal colonic tissues was fixed in 2.5% glutaraldehyde and 2% osmic acid. After dewaxing and rehydration, the embedded tissue was cut into ultrathin sections (thickness 60–70 nm), and then stained with uranium acetate and lead citrate. Autophagy was observed by transmission electron microscopy (Philips, Eindhoven, The Netherlands).

### Statistical Analysis

SPSS19.0 software was used to analyze the data of each group, and the results were presented as mean ± SD. All experiments were repeated at least three times. The student’s t test or ANOVA multiple comparisons obtain the statistical significance of differences between groups in GraphPad Prism 8.0 (GraphPad Software, La Jolla, CA), with *p* < 0.05 considered as significant.

## Results

### Integrative Pharmacological Analysis

A total of 60 overlapping targets were obtained from ETCM compound target database and Drugbank and GeneCards disease gene database, and disease gene-drug target network was constructed by Cytoscape software (Figure 1B). GO enrichment analysis showed that XLP putative targets were frequently involved in Positive regulation of autophagy, Epithelial cell development, Regulation of response to wounding, and other biological processes (Figure 1C). Pathway enrichment analysis showed that XLP putative targets involved pathway including in MAPK signaling pathway, p53 signaling pathway, and PI3K-Akt signaling pathway (Figure 1D).

### XLP Improved the Symptoms of DSS-Induced Colitis in Mice

The components of XLP were measured by LC-MS/MS (Figures 2B–E). As shown in Table 3, a total of five constituents in XLP: berberine (C20H18NO4), jatrorrhizine (C20H20NO4), costunolide (C15H20O2), coptisine (C19H14ClNO4+), and palmatine (C21H22ClNO4). To evaluate the protection of XLP on UC, we established the mice model via feeding with 3% DSS solution for consecutive 7 days (Figure 2A). Compared with control group, mice in DSS group significantly lost their weights (Figure 3A) and had a dramatic increase in DAI scores (Figure 3B). Moreover, DSS mice had shorter colons than control animals (Figure 3C). These results suggesting that the DSS treatment resulted in symptoms similar to that of clinical, which characterized with colonic edema, presence of gross bleeding and alterations in stool consistency. However, mice in 5-ASA and XLP (1.6, 3.2 g/kg) groups gradually restored their body weights, DAI scores, and colon length decreased.

**TABLE 3:** LC-MS/MS data for the Xianglian pill.

Steroid	Molecular weight (Da)	Precursor ion	Productions (ESI+)	Declustering potential	Collision energy
Berberine	336.36	336.40	319.7/277.8	133/133	31/46
Jatrorrhizine	338.38	338.30	321.7/280.1	150/150	46/55
Costunolide	232.3	233.2	105.1/145.3	96/96	32/31
Coptisine	337.2	319.5	292.2/234.0	105/105	39/51
Palmatine	352.4	351.6	335.8/294.1	120/120	31/50

**FIGURE 3:** Xianglian pill alleviated DSS-induced acute colitis in mice. **(A)** Body weight of mice in each group were monitored from day 1 to day 7. **(B)** Disease activity index of mice in each group were calculated from day 1 to day 7. **(C)** Mice were sacrificed and colonic tissues were collected and measured on day 8. **(D)** Representative hematoxylin and eosin staining images of colon tissues from each group were performed and observed under a microscope (upper panel ×100 and lower panel ×200). Histological scores of colons were calculated. **(E)** The levels of TNF-α, IL-1β, IL-6, IL-8, IL-17, and INF-γ in colon tissues from mice were measured by enzyme linked immunosorbent assay. **(F)** Detection of MPO activity and levels of NO and iNOS in colon tissues from mice were measured. *p < 0.05, **p < 0.01 vs. control group, #*p* < 0.05, ##*p* < 0.01 vs. DSS group.

### XLP Attenuated DSS-Induced Colon Injury in Mice

In order to further evaluate the protective effects of XLP on DSS induced colitis, we analyzed the histopathology of colon tissue. As shown in Figure 3D, DSS induced a severe damage of colon tissues, such as erosion of lamina propria mucosa, decrease of glandular cells and leukocyte infiltration. Oral administration of 5-ASA and XLP significantly reduced the pathological changes of colon tissue induced by DSS. The histological score further confirmed the protective effect of XLP on DSS mice, among which the high dose group of XLP had the best effect.

### XLP Suppressed DSS-Induced Expression of Inflammatory Responses in Colon

Next, the concentrations of pro-inflammatory cytokines in colon tissues were measured. As shown in Figure 3A, DSS-induced markly upregulated the concentrations of TNF-α, IL-1β, IL-6, IL-8, IL-17, and INF-γ. However, these cytokines were significantly suppressed by 5-ASA and XLP treatment. Similar to the pro-inflammatory cytokines, the results for MPO activity and levels of NO and iNOS in the colon tissues were significantly elevated in the DSS group. Nevertheless, 5-ASA and XLP oral administration alleviated the DSS-induced production of MPO, NO and iNOS in the colon (Figures 3E,F).

### XLP Attenuated Epithelial Barrier Function of DSS-Induced Colitis in Mice

The expressions of Claudin-1 and ZO-1 were detected by immunofluorescence, western blot and qRT-PCR, respectively. Immunohistochemistry staining showed that the immunoreactivity of Claudin-1 and ZO-1 in the colon tissues were significantly inhibited by DSS. However, stronger immunoreactivity was observed in the 5-ASA and XLP group than that in the DSS group (Figure 4A). Meanwhile, the results shown that oral administration of 5-ASA and XLP significantly increased the protein expression levels of Claudin-1 and ZO-1 in the colon tissues when compared to the DSS group by western blot (Figure 4B). These results were also confirmed by qRT-PCR, the mRNA expressions of Claudin-1 and ZO-1 were clearly decreased after DSS intervention, while Claudin-1 and Zo-1 mRNA expressions were significantly increased in 5-ASA and XLP compared with the DSS group (Figure 4C).

**FIGURE 4:** Xianglian pill attenuated epithelial barrier function of DSS-induced colitis in mice. **(A)** Colon tissues were stained with claudin-1 or zonula occludens-1 (red) and nuclei-stained with DAPI (blue). Fluorescence images were captured using a fluorescence microscope (×200). **(B)** Expression of claudin-1 or zonula occludens-1 in colon tissues were detected by western blot and data were expressed as fold change in protein expression normalized to β-actin expression. **(C)** Expression of claudin-1 or zonula occludens-1 mRNA in colon tissues were detected by quantitative real-time PCR and data were expressed as relative mRNA expression normalized to GAPDH expression, with respect to the control group. *p < 0.05, **p < 0.01 vs. control group, #*p* < 0.05, ##*p* < 0.01 vs. DSS group.

### XLP Enhanced Autophagy of DSS-Induced Colitis in Mice

The results of TEM showed that there were huge autophagosomes in colon tissue of control group, which indicated that the autophagy degree of colon cells was higher under normal conditions. While almost invisible autophagic vacuoles could be observed after oral administration of DSS. Treatment of 5-ASA and XLP increased the number of autophagosomes in DSS-treated colon tissue (Figure 5A). Additionally, treatment with 5-ASA and XLP markedly elevated the expression of Beclin-1 and the ratio of LC3BII/LC3BI in colitis colon tissue (Figure 5B).

**FIGURE 5:** Xianglian pill enhanced autophagy by blocked the activation of PI3K/Akt/mTOR pathway in DSS-induced colitis mice. **(A)** Autophagosomes in colon tissue from each group were detected and observed under a transmission electron microscopy (×5000). **(B)** Expression of Beclin-1 and LC3B in colon tissues were detected by western blot and data were expressed as fold change in protein expression normalized to β-actin expression or the ratio of LC3BII/LC3BI. **(C)** Expression of PI3K, p-Akt, Akt, p-mTOR, and mTOR in colon tissues were detected by western blot and data were expressed as fold change in protein expression normalized to β-actin expression. *p < 0.05, **p < 0.01 vs. control group, #*p* < 0.05, ##*p* < 0.01 vs. DSS group.

### XLP Blocked the Activation of PI3K/Akt/mTOR Pathway in DSS-Induced Colitis in Mice

Moreover, PI3K/Akt/mTOR signaling pathway, which XLP target genes involved in, has been implicated in the pathogenesis of UC, as well as autophagy and proinflammatory cytokine overproduction. In the current study, oral administration of DSS dramatically elevated the expression of PI3K and phosphorylation of Akt and mTOR in colon tissue, whereas this abnormal elevation could be reversed by treatment with 5-ASA and XLP respectively (Figure 5C).

### Inhibition of Autophagy Attenuates the Positive Effect of XLP on DSS-Induced Colitis in Mice

Next, we examined whether autophagy is crucial for the protective effect of XLP. The autophagy inhibitor 3-MA (10 mg/kg, administered intraperitoneally) was added as a pretreatment before the administration of XLP (3.2 g/kg, administered orally) could significantly reduce the autophagy promoting effect of XLP in UC mice model (Figure 6A). HE staining showed that the beneficial effects of XLP were attenuated, including colon inflammation, disease activity index, and weight loss (Figures 6B–D). Furthermore, pretreatment with 3-MA attenuated the reduction in pro-inflammatory cytokines and epithelial barrier function in the colon in XLP-treated colitis mice (Figures 6E,F).

**FIGURE 6:** Inhibition of autophagy attenuates the positive effect of XLP on DSS-induced colitis in mice. **(A)** Expression of Beclin-1 and LC3B in colon tissues were detected by western blot. **(B)** Representative hematoxylin and eosin staining images of colon tissues from each group were performed and observed under a microscope (upper panel ×100 and lower panel ×200). Histological scores of colons were calculated. **(C)** Disease activity index of mice were calculated. **(D)** Body weight of mice were monitored. **(E)** The levels of TNF-α, IL-1β, IL-6, IL-8, IL-17, and INF-γ in colon tissues were measured by enzyme linked immunosorbent assay. **(F)** Colon tissues were stained with claudin-1 or zonula occludens-1 (red) and nuclei-stained with DAPI (blue). Fluorescence images were captured using a fluorescence microscope (×200). *p < 0.05, **p < 0.01 vs. DSS group, #*p* < 0.05, ##*p* < 0.01 vs. XLP group.

## Discussion

UC is an inflammatory disease of the colon associated with the formation of ulcers and recurring inflammation. Even now, the exact mechanisms of are still not clearly understood, treatment strategies for UC are limited. The goal of for UC treatment is divided into induction of remission and maintenance of remission according to the clinical activity and the extent of diseases. Currently, glucocorticoids, aminosalicylic acid preparations and immunosuppressants are the three major kinds of agents for the clinical treatment of UC (Hauso et al., 2015; Salice et al., 2019). However, the numerous side effects of these drugs greatly restrict their clinical application. Therefore, it is urgent to develop a new therapeutic strategy with higher efficacy and less side effects to treat UC (Ung et al., 2014). XLP has been widely used in the treatment of UC in China, but the underlying mechanism remains unclear. In this study, the main ingredients of XLP were determined by LC-MS/MS. The results showed that the main ingredients of XLP included berberine, jatrorrhizine, costunolide, coptisine and palmatine. Among these constituents, berberine, palmatine and costundide have been proved to have anti-inflammatory effects in the treatment of UC through different or similar mechanisms (Mai et al., 2019; Zhu et al., 2019; Xie et al., 2020). Currently, we demonstrated the role of XLP, a classical TCM formulation, in regulating intestinal mucosal inflammation, epithelial barrier function, and autophagy in a DSS-induced colitis mouse model. To our knowledge, this is the first integrative pharmacology-based approach to predict the potential target of XLP and demonstration of the XLP effect on experimental acute colitis.

In the current study, we established a UC model by using oral administration of 3% DSS for 7 days. In which, XLP administration markedly prevented body weight loss, DAI elevation, colon length shortening. In addition, XLP can significantly relieved the colon injury caused by DSS. It is understood that persistent chronic inflammation lead to severe injury of intestinal mucosa, and unlimited production of proinflammatory cytokines is one of the most significant characteristics of uncontrolled inflammation during UC (Park et al., 2017). The present results showed that XLP significantly suppressed the contents of TNF-α, IL-1β, IL-6, IL-8, IL-17, and INF-γ, which were considered to be valuable targets for the treatment of inflammatory diseases (Yamamoto-Furusho, 2018). Moreover, it is generally known that the elevated activity of MPO and iNOS mediated excessive production of NO are considered as inflammatory biomarkers, which trigger the tissue damage, activity of neutrophils and release of pro-inflammatory cytokines in UC (Soufli et al., 2016; Aratani, 2018). And these abnormal increased could be alleviated by XLP in dose-dependent manner in the present study.

It is generally considered that epithelial barrier is the first line defense of mucosal immune system, which provides physical isolation between host immune cells and external stimuli (Camilleri et al., 2012; Ordas et al., 2012). The dysfunction of epithelial barrier leads to the migration of intestinal microbiota and the enhancement of immune system, and further induces inflammation (Merga et al., 2014; Vindigni et al., 2016). Although it is still controversial whether the Impaired epithelial barrier function is a result of chronic inflammation or precursor of UC, it is established that epithelial barrier dysfunction is a common feature of all UC patients (Lechuga and Ivanov, 2017). In the present study, our results indicated that the expression levels of claudin-1 and ZO-1 proteins and mRNAs in the intestinal tissues of DSS-induced mice were significantly downregulated, which was similar to the previous results. XLP restored epithelial mechanical barrier by elevating the expression of claudin-1 and ZO-1 in intestinal tissue in a dose-dependent manner. These results suggested that the restoration of intestinal epithelial barrier function may be part of the mechanism of XLP in inhibiting inflammation.

Autophagy is a conserved process in eukaryotes during evolution, via which cytoplasmic materials in lysosomes are degraded and is involved in many chronic inflammatory diseases (Mizushima and Komatsu, 2011; Nguyen et al., 2013). Autophagy plays a dominant role in the maintenance of intestinal homeostasis, epithelial barrier integrity, anti-microbial defense, and mucosal immune response in UC (Mizushima, 2018). Increasingly evidences support that dysregulation of the autophagy process causes disruption of several aspects of the intestinal epithelium and the immune system that can lead to an inappropriate immune response and subsequent inflammation (Sun et al., 2015; Haq et al., 2019; Wu et al., 2019). In addition, autophagy was reported to regulate intestinal barrier function by regulating lysosomal degradation of tight-junction proteins (Nighot et al., 2015). Our results reveled that XLP promoted DSS-induced autophagy inhibition. Furthermore, blocking autophagy via intraperitoneal injection of 3-MA eliminated the protective effects of XLP. These results indicate that autophagy at least partially contributes to the improved effect of XLP in UC model. PI3K/Akt/mTOR pathway is responsible for the overproduction of pro-inflammatory cytokines and mediators, as well as the main upstream regulator of autophagy (Anderson and Wong, 2010; Li et al., 2012; Bento et al., 2016). In the current study, oral administration of DSS dramatically elevated the expression of PI3K and phosphorylation of Akt and mTOR in colon tissue, whereas this abnormal elevation could be reversed by treatment with XLP.

In conclusion, XLP can alleviate DSS-induced acute colitis in mice, including inhibition the secretion of pro-inflammatory cytokines and repairing the dysfunction of intestinal epithelial barrier. The underlying mechanism may be that XLP promote autophagy by blocking the activation of PI3K/Akt/mTOR signaling pathway.

## Data Availability Statement

The raw data supporting the conclusions of this article will be made available by the authors, without undue reservation.

## Ethics Statement

The animal study was reviewed and approved by Ethics Committee of Heilongjiang Academy of Traditional Chinese Medicine.

## Author Contributions

Conceived and designed the experiments: BW, XY, and ZG. Performed the experiments: BW, XY, ZG, and LY. Analyzed and interpreted the data: BW, XY, JZ, and QZ. Drafted the paper and revised it critically for important intellectual content: BW and XY.

## Funding

This study received funding from the Natural Science Foundation of Heilongjiang Province (LH2019H095), Research project of Heilongjiang Health Committee (2020-291). Research project of traditional Chinese medicine of Heilongjiang Province (ZHY19-062, ZHY2020-041).

## Conflict of Interest

The authors declare that the research was conducted in the absence of any commercial or financial relationships that could be construed as a potential conflict of interest.
